# Edge-Preserving Median Filter and Weighted Coding with Sparse Nonlocal Regularization for Low-Dose CT Image Denoising Algorithm

**DOI:** 10.1155/2021/6095676

**Published:** 2021-07-26

**Authors:** Quan Yuan, Zhenyun Peng, Zhencheng Chen, Yanke Guo, Bin Yang, Xiangyan Zeng

**Affiliations:** ^1^School of Electronic Engineering and Automation, Guilin University of Electronic Technology, Guilin 541004, Guangxi, China; ^2^Xi'an Tapo Primary School, Chang'an District, Xi'an 710119, Shaanxi, China; ^3^School of Mathematics and Computing Science, Guilin University of Electronic Technology, Guilin 541004, Guangxi, China

## Abstract

The impulse noise in CT image was removed based on edge-preserving median filter algorithm. The sparse nonlocal regularization algorithm weighted coding was used to remove the impulse noise and Gaussian noise in the mixed noise, and the peak signal-to-noise ratio (PSNR) and structural similarity index (SSIM) were calculated to evaluate the quality of the denoised CT image. It was found that in nine different proportions of Gaussian noise and salt-and-pepper noise in Shepp-Logan image and CT image processing, the PSNR and SSIM values of the proposed denoising algorithm based on edge-preserving median filter (EP median filter) and weighted encoding with sparse nonlocal regularization (WESNR) were significantly higher than those of using EP median filter and WESNR alone. It was shown that the weighted coding algorithm based on edge-preserving median filtering and sparse nonlocal regularization had potential application value in low-dose CT image denoising.

## 1. Introduction

CT images are susceptible to the interference of quantum noise and electronic noise of detectors and other noises during the acquisition process, which causes the quality of reconstructed images to decrease, which in turn affects the diagnosis of diseases by doctors [1]. Under normal circumstances, the scan dose is proportional to the sharpness of the CT image. However, CT radiation dose is accumulated throughout the life, and multiple CT scans will increase the risk of cancer [2, 3]. Low-dose CT scan can reduce the radiation dose of patients, reduce equipment damage, reduce costs, and is conducive to the general investigation and cure of certain diseases [4]. However, the reduction of low-dose CT tube current leads to rapid degradation of projection data. After traditional algorithms are reconstructed, there are still obvious noises and artifacts in the CT reconstructed image, which seriously affects the credibility of the doctor's diagnosis. Low-dose CT scan technology is unable to give full play to its accurate diagnostic efficacy in clinical practice [5]. There may be some isolated impulse noise points in some areas of low-dose CT images. After these isolated impulse noise points are filtered, the CT image data is distributed in the form of Gaussian noise [6]. Due to the complexity of the distribution of noise and artifacts in low-dose CT images, it is difficult to establish a suitable and accurate prior model of noise in the image domain reconstruction method. The image preprocessing is complex, and the calculation is large, which affects the real-time clinical application of CT. The postprocessing method is a method that is directly applied to the reconstructed low-dose CT image to improve its image quality [7]. The method is simple and easy to implement and has good compatibility with existing CT equipment.

According to the sparse representation theory, the differences in the learning dictionary caused by individual differences and differences in tissues and organs in CT images are very small [8]. Chen et al. [5] improved the reconstruction quality of low-dose CT images with a sparse image reconstruction method. Cui et al. [9] proposed a learning method based on morphological component analysis, which can automatically generate an adaptive discriminant dictionary and effectively suppress the artifacts of low-dose CT images under the framework of sparse representation. Jiang et al. [10] proposed a denoising algorithm based on weighted coding and sparse nonlocal regularization (WESNR), which simultaneously removes impulse noise and Gaussian noise through soft impulse pixel detection. The principal component analysis (PCA) dictionary was used to encode image blocks, and the coding residuals were weighted to suppress the heavy tail of the distribution. The image sparse prior and nonlocal self-similarity prior were merged into a single nonlocal sparse regularization term, which enhances the stability of weighted coding. However, when this method was applied to low-dose CT image denoising, details were lost, and edges were destroyed. A variety of edge preservation filters can solve the problem of incorrect removal of edges and lines in the image denoising process. The feature of edge-preserving filtering is that it can extract the spatial constraint factors of the edge information in the reference image to process the original image, thereby smoothing and edge-preserving it. Among them, edge-preserving median filter (EP median filter) has a good performance in terms of operation speed and edge protection [11]. However, the edge-preserving filtering algorithm is not effective for mixed noise and noise with low signal-to-noise ratio.

In this exploration, a denoising algorithm based on EP median filter and WESNR is proposed, which can remove the mixed noise of low-dose CT image and preserve the edge information of the image.

## 2. Algorithm Based on WESNR and EP Median Filter

### 2.1. Mixed Noise Model

For image *x* with size *m* × *n*, *x*_*i*,*j*_ is the gray value at (*i*, *j*), and *y* is set as the observed image of image *x*. For adding Gaussian noise, the pixels *y*_*i*,*j*_ in *y* are defined as *y*_*i*,*j*_=*x*_*i*,*j*_+*v*_*i*,*j*_, where *v*_*i*,*j*_ is the independent and identically distributed noise; for the salt-and-pepper noise, [*d*_min_, *d*_max_] represents the dynamic range of *y* pixels in the observation image, and the probability of salt-and-pepper noise is *s*, 0 ≤ *s* ≤ 1. Then, the probability of *y*_*i*,*j*_=*d*_min_ is *s*/2, and the probability of *y*_*i*,*j*_=*d*_max_ is *s*/2. Therefore, the observation image mixed with Gaussian noise and salt-and-pepper noise can be described as follows:

(1) $$\begin{array}{c} y_{i,j}=\left\{\begin{array}{cc} d_{\min}, & \text{the probability is }\frac{\text{s}}{2},\\ d_{\max}, & \text{the probability is }\frac{\text{s}}{2},\\ x_{i,j}+v_{i,j}, & \text{the probability is }1-s. \end{array}\right. \end{array}$$

### 2.2. EP Median Filter Algorithm

The pixel at (*i*, *j*)(3 ≤ *i* ≤ *m* − 2,3 ≤ *j* ≤ *n* − 2) in image *y* has the neighborhood of 5 × 5 in Figure 1. If (*i*, *j*) is a point in a flat area, most of the gray values of 24 pixels in its neighborhood should be close to it. Even if there are few noise points, it can be set to less than one-fourth; that is, the number *t*_*i*,*j*_ of absolute values of gray value difference greater than a certain threshold *T* is less than or equal to 6; if (*i*, *j*) is an edge point, about half of the gray values of the 24 pixels in its neighborhood should be close to it, and the other half should have a large difference with it; that is, the number *t*_*i*,*j*_ of gray values whose absolute value is greater than a certain threshold *T* should be about 12; if (*i*, *j*) is a noise point, most of the gray values of the 24 pixels in its neighborhood should not be close to it. It can be set as no less than three-fourths; that is, the number *t*_*i*,*j*_ of absolute values of gray value difference greater than a certain threshold value *T* is greater than or equal to 18.

The standard deviation of image *y* is taken as the threshold *T*; that is,

(2) $$\begin{array}{c} T=\sqrt{\frac{\sum_{i=1}^{m}\sum_{j=1}^{n}{\left(y_{i,j}-\bar{y}\right)}^{2}}{m\cdot n}}, \end{array}$$

where $\bar{y}$ is the mean value of all gray values of image *y*; that is,

(3) $$\begin{array}{c} \bar{y}=\sqrt{\frac{\sum_{i=1}^{m}\sum_{j=1}^{n}\left(y_{i,j}\right)}{m\cdot n}}, \end{array}$$

Based on the above assumption, (*i*, *j*)(3 ≤ *i* ≤ *m* − 2,3 ≤ *j* ≤ *n* − 2) can be divided into points in flat area, edge points, and noises.

① *t*_*i*,*j*_ ≤ 6, (*i*, *j*) is the point of the flat area.
② 6 < *t*_*i*,*j*_ < 18, (*i*, *j*) is the edge point.
③ *t*_*i*,*j*_ ≥ 18, (*i*, *j*) is the noise.

When (*i*, *j*) is noise, the gray value at (*i*, *j*) of the original image is replaced by the mean value of *y*_*i*,*j*_, *y*_*i*,*j*−1_, *y*_*i*−1,*j*_, *y*_*i*+1,*j*_, *y*_*i*,*j*+1_, *y*_*i*−1,*j*−2_, *y*_*i*+1,*j*−2_, *y*_*i*−2,*j*−1_, *y*_*i*+2,*j*−1_, *y*_*i*−2,*j*+1_, *y*_*i*+2,*j*+1_, *y*_*i*−1,*j*+2_, and *y*_*i*+1,*j*+2_. The pixels participating in the assignment and their gray values are the shadow parts in Algorithm 1, and the mean value is *a*_*i*,*j*_; that is,

(4) $$\begin{array}{c} a_{i,j}=\frac{\left(y_{i,j}+y_{i,j-1}+y_{i-1,j}+y_{i+1,j}+y_{i,j+1}+y_{i-1,j-2}+y_{i+1,j-2}+y_{i-2,j-1}+y_{i+2,j-1}+y_{i-2,j+1}+y_{i+2,j+1}+y_{i-1,j+2}+y_{i+1,j+2}\right)}{13}. \end{array}$$

The gray values of all the pixels in (*i*, *j*)(*i* ≤ 2,  or *i* ≥ *m* − 2,  or *j* ≤ 2,  or *j* ≥ *n* − 2) are not modified, the gray values of the points in the flat area and the edge points in (*i*, *j*)(3 ≤ *i* ≤ *m* − 2,  3 ≤ *j* ≤ *n* − 2) are not modified, and the noise in (*i*, *j*)(3 ≤ *i* ≤ *m* − 2,  3 ≤ *j* ≤ *n* − 2) is replaced by the value of *a*_*i*,*j*_, so that the gray values of the pixels in the (*i*, *j*) position of the denoised image are *y*_*i*,*j*_′. There is

(5) $$\begin{array}{c} y_{i,j}^{\prime }=\left\{\begin{array}{cc} y_{i,j}, & i\leq 2,\text{ or }i\geq m-1,\text{ or }j\leq 2\text{ or }j\geq n-1,\\ y_{i,j}, & 3<i<m-2,\;3<j<n-2\text{ and }t_{i,j}<18,\\ a_{i,j}, & 3<i<m-2,\;3<j<n-2\text{ and }t_{i,j}\geq 18. \end{array}\right. \end{array}$$

If *y*′ is the image with size *m* × *n* and the gray value at (*i*, *j*) is *y*_*i*,*j*_′, *y*′ is the denoised image of observation image *y* by EP median filter algorithm.

### 2.3. WESNR Algorithm

For image *x*, *x*_*i*_=*R*_*i*_*x* ∈ *R*^*n*′^ represent the image block of size $\sqrt{n^{\prime }}\times \sqrt{n^{\prime }}$, where *R*_*i*_ is the matrix vector. Based on the sparse representation theory, the image block is sparse-coded through the overcomplete dictionary Φ=[*ϕ*_1_; *ϕ*_2_; …; *ϕ*_*n*_] ∈ *R*^*n*′×*m*′^, so that *x*_*i*_=Φ*α*_*i*_, where *α*_*i*_ is the sparse coding vector of nonzero matrix. The results are as follows:

(6) $$\begin{array}{c} x=\Phi \alpha , \end{array}$$

where *α* is the set of all sparse coding vectors *α*_*i*_.

The traditional sparse representation denoising algorithm can be expressed as

(7) $$\begin{array}{c} \hat{\alpha }=\underset{\alpha }{\arg\min}{\left\|y-\Phi \alpha \right\|}_{2}^{2}+\lambda R\left(\alpha \right), \end{array}$$

where *R*(*α*) is a regularization term corresponding to *α* and *λ* is a regularization parameter.

To make the distribution of data fitting residuals more regular, data residuals are weighted [12]. A new loss function is used, and the following mixed noise removal model is obtained:

(8) $$\begin{array}{c} \hat{\alpha }=\underset{\alpha }{\arg\min}{\left\|W^{\left(1/2\right)}\left(y-\Phi \alpha \right)\right\|}_{2}^{2}+\lambda R\left(\alpha \right), \end{array}$$

where *W* is a diagonal weight matrix with diagonal elements.

Image block *x*_*i*_ and its nonlocal prediction are encoded by a given dictionary *ϕ*_*i*_; that is, *x*_*i*_=*ϕ*_*i*_*α*_*i*_ and ${\hat{x}}_{i}=\phi_{i}\mu_{i}$, and then the encoding coefficients *x*_*i*_ and *μ*_*i*_ are similar. Therefore, ∑_*i*_‖*α*_*i*_ − *μ*_*i*_‖_*l*_*p*__ is used as the regularization term and applied to the above equation. There is

(9) $$\begin{array}{c} \hat{\alpha }=\underset{\alpha }{\arg\min}{\left\|W^{\left(1/2\right)}\left(y-\Phi \alpha \right)\right\|}_{2}^{2}+\lambda \sum_{i}{\left\|\alpha_{i}-\mu_{i}\right\|}_{l_{p}}, \end{array}$$

where *l*_*p*_ (*p*=1 or *p*=2) is the *l*_*p*_ norm. *l*_1_ is chosen as the norm. The model is as follows:

(10) $$\begin{array}{c} \hat{\alpha }=\underset{\alpha }{\arg\min}{\left\|W^{\left(1/2\right)}\left(y-\Phi \alpha \right)\right\|}_{2}^{2}+\lambda \sum_{i}{\left\|\alpha_{i}-\mu_{i}\right\|}_{1}, \end{array}$$

where *W* is a diagonal weighted matrix whose element *W*_*ii*_ will be determined automatically. The coding residual *e*_*i*_ can be used to determine the weight *W*_*ii*_, and the strength of *W*_*ii*_ is inversely proportional to that of *e*_*i*_. *W*_*ii*_ ∈ [0,1] is set. *W*_*ii*_ is determined as

(11) $$\begin{array}{c} W_{ii}=\exp\left(-ae_{i}^{2}\right). \end{array}$$

Iterative reweighting is used to solve the problem. *V* is set to a diagonal matrix and initialized as an identity matrix. In *k*+1 times of iteration, each element of *V* is updated as follows:

(12) $$\begin{array}{c} V_{ii}^{\left(k+1\right)}=\frac{\lambda }{{\left({\left(\alpha_{i}^{\left(k\right)}-\mu_{i}\right)}^{2}+\varepsilon^{2}\right)}^{\left(1/2\right)}}, \end{array}$$

where *ε* is a scalar and *α*_*i*_^*k*^ is the *i*-th element of the coding vector *α* in the *k*-th iteration. The sparse coding *α* is updated by the following function:

(13) $$\begin{array}{c} {\hat{\alpha }}^{\left(k+1\right)}={\left(\Phi^{T}W\Phi +V^{\left(k+1\right)}\right)}^{-1}\left(\Phi^{T}Wy-\Phi^{T}W\Phi \mu \right)+\mu . \end{array}$$

A set of local PCA dictionaries are learned from natural images, and the model can be solved by iteratively updating *W* and *α*. The update of *W* depends on the coding residual *e*, and the adaptive median filter is selected for *y* to get an initial image *x*^(0)^. Then, *e* is initialized to

(14) $$\begin{array}{c} e^{\left(0\right)}=y-x^{\left(0\right)}. \end{array}$$

The above optimization is repeated for the subproblem until the iteration stop condition is satisfied. When there is no significant change in the solution of continuous iteration or the corresponding objective function value, that is, when the difference norm between two continuous iterative solutions is less than the given positive norm, the algorithm stops, or when the running time exceeds the upper limit, the iterative process stops. In this exploration, *t*=‖Φ*α*^(*k*+1)^ − Φ*α*^(*k*)^‖_2_/‖Φ*α*^(*k*)^‖_2_ < *τ* is regarded as the termination condition. The obtained image is the denoised image of the observed image *y* by the WESNR algorithm.

### 2.4. Denoising Algorithm Based on EP Median Filter and WESNR

The general denoising algorithm will inevitably lose the details of the image. In particular, for the image with more lines, it will cause the blurring of the visual effect. In order to avoid the situation that the lines and edges of objects in the image are eliminated by mistake in the process of denoising, EP median filter algorithm distinguishes lines or edges from noise in advance, which has good performance in image details and edge preservation. However, EP median filter algorithm is only suitable for the removal of impulse noise in the image, and it does not perform well in the removal of other noises or mixed noises. When low-dose CT images with complex noise are processed, the phenomenon of incomplete noise removal will appear.

WESNR algorithm encodes each noise contaminated block, which can remove the mixed noise of impulse noise and Gaussian noise at the same time. However, for low-dose CT image denoising, when WESNR algorithm is used directly, there will be loss of details and edge damage.

In order to achieve the purpose of removing mixed noise in the process of low-dose CT image denoising without destroying the details and edges, EP median filter algorithm is combined with WESNR algorithm. First, the points in the center region of the noisy image *y* are classified into points in flat areas, edge points, and noise points. The points in the flat area, the edge points, and the points outside the central area are not replaced. The noise in the central region is replaced by the mean value of the gray value of 13 pixels around it to get image *y*′ after the first step. Then, *y*′ is input into WESNR algorithm as noisy image, and local PCA dictionary is selected to iterate the target problem, subproblem, and parameters. When the preset termination condition is satisfied, image *y*^″^ is the result of the denoising algorithm based on EP median filter and WESNR. Algorithm 1 shows the flow of the algorithm.

The steps of denoising algorithm based on EP median filter and WESNR are as follows.

## 3. Experiment

In addition to the visual effect comparison, the following numerical criteria are given: peak signal-to-noise ratio (PSNR) and structural similarity (SSIM). PSNR is the most commonly used objective index to evaluate image quality, which is an objective description of the degradation degree of an image. The higher the value of PSNR is, the closer it is to the original image. SSIM is mainly used to measure the similarity between the original image and the restored image. The higher the SSIM, the higher the image quality [13].

### 3.1. Shepp-Logan Head Model Experiment

The Shepp-Logan head model of 256 *∗* 256 is selected as the experimental object. This model was proposed by Shepp and Logan in 1974 [14]. The image is composed of 10 ellipses with different positions, sizes, directions, and densities. Different gray value of ellipse can simulate attenuation coefficient of different tissues, and Shepp-Logan head model can simulate human head sectional image well. In Shepp-Logan image, the mixed noise with different proportions of Gaussian noise and salt-and-pepper noise are added, respectively. EP median filter algorithm, WESNR algorithm, and the algorithm proposed in this exploration are used to denoise the image. The reconstruction effect and numerical comparison of various algorithms under nine kinds of noise are listed, as shown in Figure 2 and Table 1. The bold fonts in the table indicate the advantages of the algorithm.

The experimental results show that, for nine kinds of Shepp-Logan images with different proportions of Gaussian noise and salt-and-pepper noise, the reconstruction effect and numerical comparison of the proposed denoising algorithm based on EP median filter and WESNR are better than those of EP median filter algorithm and WESNR algorithm alone. Moreover, the proposed algorithm has the advantages of good edge preservation and good effect of removing mixed noise.

### 3.2. Low-Dose Brain CT Simulation Image

A brain CT image with 512 *∗* 512 pixels is selected as the experimental object. Different proportions of Gaussian noise and salt-and-pepper noise are added to simulate the image output effect of low-dose CT. The reconstruction effect and numerical comparison of various algorithms under nine kinds of noise are listed, as shown in Figure 3 and Table 2. The bold fonts in the table indicate the advantages of the algorithm.

The experimental results show that, for nine kinds of simulated low-dose brain CT images with different proportions of Gaussian noise and salt-and-pepper noise, the proposed denoising algorithm based on EP median filter and WESNR outperforms EP median filter algorithm and WESNR algorithm alone in terms of reconstruction effect and numerical comparison. Moreover, the proposed algorithm has the advantages of good details and edge preservation and good effect of removing mixed noise.

## 4. Conclusion

In this exploration, a new low-dose CT image denoising algorithm is proposed. According to the characteristics of low-dose CT image and noise, this algorithm is to combine EP median filter with WESNR. The experimental results show that the algorithm proposed in this exploration has a good ability to suppress the mixed noise in low-dose CT images, and the edge information is well preserved. However, this study still has some shortcomings. The proposed method is not compared with other related low-dose CT image noise reduction algorithms, and its effect on low-dose CT image noise reduction needs further study. In the future work, we will continue to compare it with related algorithms to clarify the value of this algorithm in low-dose CT images for noise reduction. In short, the algorithm of this research has a significant effect on denoising mixed noise in low-dose CT images.

## Figures and Tables

**Figure 1:** Gray value of (*i*, *j*) and its neighborhood Algorithm 1 Pixels participating in *a*_*i*,*j*_′ assignment and their gray values.

**Figure 2:** Denoising effect of different methods on Shepp-Logan image. (a) The original Shepp-Logan image. (b) The Shepp-Logan image after adding mixed noise *σ*=5,  *ρ*=20%. (c) Denoising effect of EP median filter algorithm. (d) Denoising effect of WESNR algorithm. (e) Denoising effect of the algorithm proposed in this exploration.

**Figure 3:** Denoising effect of different methods on brain CT image. (a) The original image of brain CT. (b) Simulated low-dose brain CT images with mixed noise of *σ*=5,  *ρ*=20%. (c) Denoising effect of EP median filter algorithm. (d) Denoising effect of WESNR algorithm. (e) Denoising effect of the algorithm proposed in this exploration.

**Algorithm 1:** Flow chart of the algorithm proposed.

**Table 1:** Comparison of PSNR and SSIM of denoised Shepp-Logan image.

*σ*	*ρ* (%)	EP median filter		WESNR		The algorithm proposed in this exploration	
		PSNR	SSIM	PSNR	SSIM	PSNR	SSIM
5	10	23.25	0.5233	32.76	0.8589	33.31	0.8841
	20	19.85	0.4511	28.68	0.8341	30.01	0.9026
	30	16.78	0.3399	27.14	0.8153	27.59	0.9028

10	10	22.60	0.3337	31.22	0.6922	31.94	0.7393
	20	19.62	0.2963	29.29	0.6829	30.20	0.7766
	30	16.24	0.2192	26.43	0.6534	26.73	0.7819

20	10	20.77	0.1943	28.16	0.4816	28.96	0.5349
	20	18.28	0.1681	26.83	0.4482	27.85	0.5418
	30	15.85	0.1382	25.99	0.4413	27.38	0.5813

**Table 2:** Numerical comparison of PSNR and SSIM after denoising of simulated low-dose brain CT images.

*σ*	*ρ* (%)	EP median filter		WESNR		The algorithm proposed in this exploration	
		PSNR	SSIM	PSNR	SSIM	PSNR	SSIM
10	10	25.40	0.4115	33.87	0.5428	34.20	0.6123
	20	21.41	0.3813	31.95	0.5304	32.26	0.6757
	30	17.11	0.2933	28.68	0.5302	29.41	0.7335

20	10	22.49	0.2165	28.38	0.3950	30.00	0.4107
	20	20.11	0.1970	27.84	0.3526	29.17	0.4710
	30	16.43	0.1539	26.75	0.3376	27.79	0.5054

30	10	20.05	0.1498	25.67	0.2773	26.92	0.3162
	20	18.48	0.1337	25.14	0.2702	26.83	0.3604
	30	15.52	0.1089	24.29	0.2632	25.94	0.4110

## Data Availability

The data used to support the findings of this study are available from the corresponding author upon request.
